The article "Outcome Predictors of Percutaneous Cholecystostomy As Definitive Versus Bridging Treatment for Acute Cholecystitis" was published in 2023. Journal: Cureus.

# Outcome Predictors of Percutaneous Cholecystostomy As Definitive Versus Bridging Treatment for Acute Cholecystitis

**DOI:** 10.7759/cureus.49962

**Published:** 2023-12-05

**Authors:** Joshua Lau, Surajit Sinha

**Affiliations:** 1 Upper GI Surgery, Torbay & South Devon NHS Foundation Trust, Torquay, GBR

**Keywords:** minimally invasive interventional radiology, mortality predictor, charlson comorbidity index, definitive treatment, bridging treatment, predictive factor, cholecystostomy drain, percutaneous cholecystostomy tube, cholecystectomy laparoscopic, acute cholecystitis

## Abstract

Introduction

Percutaneous cholecystostomy (PC) is a treatment option for patients with acute cholecystitis (AC) who are too unwell, or too morbid for laparoscopic cholecystectomy (LC). Some patients have PC as a definitive treatment, whereas others have PC as a bridging treatment prior to LC. The aim of this study is to investigate patient characteristics and mortality among those who received PC as definitive treatment versus bridging treatment.

Methods

Our study retrospectively reviewed all patients treated with PC for AC from February 2019 to November 2022 at the Torbay and South Devon NHS Foundation Trust, Torquay, England. Fifty patients underwent PC for AC, with 48 patients having follow-up data available for analysis. Of these, 26 patients (54%) only received PC (definitive PC), and 22 patients (46%) later underwent LC (bridging LC).

Results

In this study, 68.8% of the patients were male, with a mean age of 76 ± 9 years. The overall mean Charlson Comorbidity Index (CCI) score was 4.96 ± 1.12, and the mean American Society of Anesthesiologists (ASA) score was 2.83 ± 0.36. The median PC drain duration was 42 days. Six patients (12.5%) had a recurrence of AC with a mean of 57 days onset after PC insertion. Twelve patients (25%) experienced PC complications: 11 (23%) were minor, involving pain or a dislodged tube, and one (2%) was major, resulting in a subhepatic abscess.

The median duration from PC insertion to LC surgery was 50.5 days. The bridging LC cohort had a 30-day and one-year mortality of 0%, while the definitive PC cohort had a 30-day mortality of 30.8% (eight patients) and a one-year mortality of 46.1% (12 patients). The bridging LC cohort compared to the definitive PC cohort had a significantly lower CCI (4.39 vs 5.57, p<0.05), and a significantly lower ASA (2.61 vs 3.04, p<0.05). The one-year survival cohort compared to the 30-day mortality cohort had significantly lower ASA (2.71 vs 3.25 p<0.05), and a non-significantly lower CCI (4.66 vs 5.86 p=0.094). The presence of negative predictive factors of respiratory dysfunction and hyperbilirubinemia had higher 30-day and 90-day mortality rates of 31.3% and 37.5%, compared to their absence of 9.4% and 21.4% respectively.

The article "Outcome Predictors of Percutaneous Cholecystostomy As Definitive Versus Bridging Treatment for Acute Cholecystitis" was published in 2023. Journal: Cureus.

Conclusion

Our results demonstrate that PC is a safe procedure with a high success rate and low complications. We showed that PC is an effective treatment option for bridging a select cohort of patients to receive a delayed LC. Furthermore, the data suggests ASA and CCI scoring can be used as clinical adjuncts to assess whether bridging patients from PC to LC is appropriate. Finally, ASA, respiratory dysfunction, and hyperbilirubinemia can be used as significant negative predictors of post-PC mortality.

## Introduction

Acute cholecystitis (AC) is a common surgical presentation. Approximately 15% of the United Kingdom’s (UK) population have gallstones, of which 20% will present with gallstone complications, including AC [1]. AC can cause severe complications such as gallbladder perforation, jaundice, and sepsis, and has a mortality of approximately 3% [2]. The gold standard of treatment of AC is laparoscopic cholecystectomy (LC), recommended by both the UK’s National Institute of Clinical Excellence (NICE) guidelines as well as the Tokyo Guidelines, and the World Society of Emergency Surgery (WSES) guidelines [3-5].

Patients who are elderly, have multiple comorbidities, or are septic from AC face higher surgical and overall mortality risks. One large retrospective UK study demonstrated that patients aged over 80 years have an 11.6% 30-day mortality and a 20.8% one-year mortality following LC for AC [6]. Negative predictive factors of neurological or respiratory dysfunction, or high bilirubin, have been identified and associated with higher surgical mortality in AC [7]. The Charlson Co-morbidity Index (CCI) score, and American Society of Anaesthesiology (ASA) scores are also predictive of surgical mortality [8]. Negative predictive factors, CCI scores, and ASA scores are all recommended by the Tokyo Guidelines 2018 for AC management to guide surgical decision-making [9]. 

Percutaneous cholecystostomy (PC) is an effective, minimally invasive treatment of AC that is recommended by NICE, WSES, and Tokyo Guidelines for patients at high risk from surgery as an alternative to AC [3-5]. PC can be used as a singular ‘definitive’ treatment for AC but has been increasingly used as a bridging treatment for a delayed LC after acute sepsis has resolved [10-12]. However, there is little evidence or guidance published to suggest which patients receiving PC for AC would benefit from a delayed LC.

In this study, we utilized the Tokyo Guidelines 2018 recommendations for patient predictive factors of organ dysfunction on presentation, as well as CCI and ASA scores for AC outcomes, to assess whether these factors were also predictive of outcomes for our patients undergoing PC as definitive versus bridging treatment for AC.

The article "Outcome Predictors of Percutaneous Cholecystostomy As Definitive Versus Bridging Treatment for Acute Cholecystitis" was published in 2023. Journal: Cureus.

## Materials and methods

Data was collected retrospectively for all patients who were treated with PC for AC from February 2019 to November 2022 at Torbay and South Devon NHS Foundation Trust, Torquay, England. All data was anonymised and approved by the local audit department, Torbay Hospital Clinical Effectiveness Department (project/approval number: i-0323).

Patients without a minimum of one year of follow-up data were excluded. Patients were divided into the 'definitive PC' cohort for those receiving PC as the sole treatment for AC and the 'bridging LC' cohort for those undergoing a delayed LC following PC treatment.

Demographic data, including age and gender, were collected. Patient CCI and ASA were calculated from their past medical history records. Neurological status was determined based on the early warning score at admission, respiratory dysfunction from oxygen requirements and respiratory rate at admission, and bilirubin from liver function tests at admission. The study also investigated the duration of PC drain and the time interval between PC and LC. The primary outcome assessed was the 30-day, 90-day, and one-year mortality. The secondary outcomes assessed were the recurrence rate of AC and PC complication rates.

Data was entered into an Excel spreadsheet (Microsoft Corporation, Redmond, Washington, United States) and analysed using IBM SPSS Statistics for Windows, Version 29.0 (Released 2022; IBM Corp., Armonk, New York, United States).

## Results

Demographics

During the study period, a total of 48 patients received PC for AC. Of these, 26 patients (54%) underwent PC as their definitive treatment, while 22 patients (46%) had PC as a bridging treatment for a delayed LC. The median duration between PC and AC was 50.5 days (Figure 1).

**Figure 1:** Definitive PC versus Bridging LC rates PC: Percutaneous Cholecystostomy; LC: Laparoscopic Cholecystectomy Data has been represented as n

Of the 48 patients, 33 (69%) were male, and 15 (31%) were female. The majority of patients (n=21; 44%) fell within the 72-80 age range. Additionally, 16 patients (33%) were above 80 years of age (Figure 2).

**Figure 2:** Overall age distribution Data has been represented as n

The mean CCI for the entire PC cohort was 4.96 (± 1.12) (Figure 3), and the mean ASA was 2.83 (± 0.35) (Figure 4).

**Figure 3:** Patient data categorised into CCI score levels CCI: Charlson Comorbidity Index Data has been represented as n

**Figure 4:** Patient data categorised into ASA score levels ASA: American Society of Anesthesiologists Data has been represented as n

Within the PC cohort, 16 patients (33%) had respiratory dysfunction, eight patients (17%) had hyperbilirubinemia (bilirubin ≥ 34 µmol/L), and two patients (4%) had both respiratory dysfunction and hyperbilirubinemia. No patients presented with neurological dysfunction (Figure 5). 

The article "Outcome Predictors of Percutaneous Cholecystostomy As Definitive Versus Bridging Treatment for Acute Cholecystitis" was published in 2023. Journal: Cureus.

**Figure 5:** Patient negative predictive factor distribution 'Respiratory' indicates respiratory dysfunction at presentation (raised respiratory rate/increased oxygen requirements); 'Bilirubin' indicates Bilirubin > 34 umol/L at presentation; 'Both' indicates both respiratory dysfunction and bilirubin > 34 umol/L at presentation. Data has been represented as n

Overall mortality

Mortality was determined to be 16.7% (eight patients) at one month and 27.9% (12 patients) at both 90 days and one year post PC insertion (Figure 6).

**Figure 6:** Cumulative patient mortality at different time points post PC insertion PC: Percutaneous Cholecystostomy Data represented as % of total patient population (n = 48)

Cholecystostomy efficacy and complications

All PC procedures were performed transhepatically and achieved a 100% success rate. The median duration of PC drain insertion was 42 days. Six patients (12.5%) treated with PC returned to the hospital with a recurrence of AC, with a median duration of 57 days following PC insertion (Figure 7).

**Figure 7:** Overall patient AC recurrence rate AC: Acute Cholecystitis Total patient population n = 48; Data represented as n and %

Fourteen patients (29%) experienced PC complications, with the most common being the falling out or dislodging of the PC tube (10 patients, 21%), followed by moderate/severe pain around the drain site in four patients (8%), and one patient (2%) developing a subhepatic abscess (Figure 8).

**Figure 8:** Patient PC complication rates and distribution PC: Percutaneous Cholecystostomy Data has been represented as n

Tubogram and acute cholecystitis recurrence

Tubograms were regularly performed on PC patients to assess both cystic and common bile duct patency. These procedures were conducted after the resolution of sepsis and before capping the drain. Out of the initial 48 patients, eight had their PC tubes fall out, four had previously undergone computed tomography/magnetic resonance cholangiopancreatography (CT/MRCP), and eight had died, leaving 28 patients who should have undergone a tubogram. Among those 28 patients, 24 (85%) appropriately received a tubogram. Of these, 15 tubograms (62.5%) showed normal biliary flow into the duodenum, six (25%) revealed either duct obstruction or gallbladder perforation, and three (12.5%) showed a dislodged PC tube (Figure 9).

The article "Outcome Predictors of Percutaneous Cholecystostomy As Definitive Versus Bridging Treatment for Acute Cholecystitis" was published in 2023. Journal: Cureus.

**Figure 9:** Tubograms performed in PC PC: Percutaneous Choleystostomy

In the normal tubogram cohort (n = 15), three patients (20%) experienced a recurrence of AC. In the dislodged/obstructed/perforated tubogram cohort (n = 9), two patients (22%) had a recurrence of AC (Figure 10).

**Figure 10:** AC recurrence in patients with normal tubogram versus abnormal tubogram AC: Acute Cholecystitis The data has been represented as n and %

Definitive PC versus bridging LC

The mortality rate of the definitive PC cohort (n = 26) was 30.8% (n = 8) at 30 days, 46.2% (n = 12) at 90 days, and remained at 46.2% at one year. Meanwhile, the mortality rate of the bridging LC cohort (n = 22) was 0% at 30 days, 90 days (Figure 11), and one year.

**Figure 11:** LC versus PC mortality rates at different time periods LC: Laparoscopic Cholecystectomy; PC: Percutaneous Cholecystostomy The data has been represented as n and %

The mean CCI score of the LC bridging cohort (n = 22) was 4.39 (± 2.3), while for the definitive PC cohort (n = 26), it was 6.3 (± 2.59). There was a statistically significant difference (p < 0.05) between the mean CCI scores of the LC and PC cohorts. Similarly, the mean ASA score of the LC bridging cohort was 2.61 (± 0.76) compared to 3.04 (± 0.62) for the definitive PC cohort. Again, there was a statistically significant difference (p < 0.05) between the mean ASA scores of the LC and PC cohorts (Figure 12).

**Figure 12:** CCI and ASA scores in LC versus PC LC: Laparoscopic Cholecystectomy; PC: Percutaneous Cholecystostomy; CCI: Charlson Co-morbidity Index; ASA: American Society Anaesthesiology Data represented as mean±SD

ASA, CCI, and negative predictive factors versus overall mortality

The mean ASA for the 'alive at one-year' cohort (n=36) was 2.71 (± 0.71), while for both the 30-day mortality cohort (n=8) and the 90-day mortality cohort (n=12), it was 3.25 (± 0.62). There was a statistically significant difference between the mean ASA of the 'alive at one-year' cohort and the 30-day and 90-day mortality cohorts (p < 0.05) (Figure 13).

**Figure 13:** Mean ASA of different mortality cohorts ASA: American Society of Anaesthesiology The data has been represented in mean±SD

The mean CCI for the 'alive at one-year' cohort (n=36) was 4.66 (± 2.27). For the 30-day mortality cohort, the mean CCI was 5.86 (± 2.53), and for the 90-day mortality cohort, it was 5.91 (± 2.15). There was a non-significant difference between the mean CCI of the 'alive at one-year' cohort and the 30-day mortality cohort (p = 0.094) (Figure 14).

**Figure 14:** Mean CCI of different mortality cohorts CCI: Charlson Co-morbidity Index The data has been represented as mean±SD

Patients with no negative predictive risk factors present on admission (no respiratory or neurological dysfunction, and no hyperbilirubinemia ≥ 34 µmol/L) (n=32) experienced a 30-day mortality of 9.4% (three patients), a 90-day mortality of 21.4% (seven patients), and a one-year mortality of 21.4% (seven patients). In contrast, patients with negative predictive risk factors present on admission (n = 16) had a 30-day mortality of 31.3% (five patients), a 90-day mortality of 37.5% (six patients), and a one-year mortality of 37.5% (six patients) (Figure 15). In the one-year survival group, compared to the 30-day mortality group, there was a lower rate of respiratory dysfunction (9.4% vs. 31.3%), but no significant difference in the presence of raised bilirubin > 34 µmol/L (17.5% vs. 12.5%).

The article "Outcome Predictors of Percutaneous Cholecystostomy As Definitive Versus Bridging Treatment for Acute Cholecystitis" was published in 2023. Journal: Cureus.

**Figure 15:** Negative predictive factors and mortality rates Negative predictive factors: respiratory dysfunction or hyperbilirubinemia The data was represented as n and %

## Discussion

The UK’s NICE guidelines, along with the European's WSES 2020 and the Tokyo Guidelines 2018, recommend LC as the preferred treatment option for AC in patients who are surgically fit [3-5]. However, patients who are comorbid or septic face significantly higher surgical risks [6]. PC is a minimally invasive option for these patients, and with an increasingly elderly and comorbid population, the incidence of PC has increased with a decrease in LC [13].

While PC has shown safety and effectiveness for AC treatment, studies such as the recent randomised controlled trial (RCT) CHOCOLATE (Laparoscopic cholecystectomy versus percutaneous catheter drainage for acute cholecystitis in high-risk patients) Trial 2018 revealed comparable mortality between PC and LC, but more biliary disease recurrence and longer hospital stays with PC [14]. This has prompted ongoing discussions about the role of interval cholecystectomy following PC, and for which patients this should be considered. Yet, very few studies have researched the indications and outcomes of this practice.

The current study aimed to investigate patient factors predicting outcomes for those receiving PC definitively versus bridging to LC. We focused on factors recommended by the Tokyo Guidelines for AC grading and mortality. As expected, our PC cohort consisted of individuals mostly above the age of 70, with multiple comorbidities, with a mean CCI of 4.96 and a mean ASA of 2.93. A recent RCT in 2020 demonstrated that patients above the age of 80, with a CCI > 5, and ASA > 3 were at very high risk of surgery [15], suggesting our PC cohort had appropriately avoided or delayed surgery. The entire PC cohort showed an average mortality of 16.7% at 30 days and 27.9% at 90 days, which is similar to a 2009 systemic review of a 15.4% mortality rate at 30 days [16], but lower than another study showing a 37.7% mortality rate at one year [17].

The article "Outcome Predictors of Percutaneous Cholecystostomy As Definitive Versus Bridging Treatment for Acute Cholecystitis" was published in 2023. Journal: Cureus.

In the current study, PC procedures had a 100% success rate, and complications were mainly minor including tube dislodgement/blockage or pain, with only one major complication of infection. This is similar to the minor complication rates cited in the literature, with the current study showing a lower major complication rate than the cited sepsis rate of 3.5-5% [18]. AC recurrence in our PC cohort was 12.5%, significantly lower than other studies, which showed 22% and 40% [17,19].

Tubograms are a fluoroscopic technique commonly used in our NHS Trust for PC patients after resolution of sepsis, or if there are issues with the drain. Theoretically, an abnormal tubogram showing bile duct obstruction or gallbladder perforation should increase the risk of recurrence of AC. However, our results show no significant difference between the 20% AC recurrence in the normal tubogram cohort compared to the 22% AC recurrence in the abnormal tubogram cohort. This would suggest that tubograms have limited use in guiding the removal of drains, which is similar to literature findings [20]. However, results may not be reliable due to the low number of AC recurrences, and also the low number of tubograms due to ERCPs and deaths precluding their need.

Of the 48 patients in total, 26 (54%) had PC as their definitive treatment and 22 (46%) had PC as bridging treatment to a delayed LC, with a median duration of 50.5 days. The bridging LC rates in the current study were similar to other studies and had a shorter duration between PC and surgery than the 116 and 144 days in those studies [21,22].

The most significant finding in our study was a 0% mortality rate at one-year post PC for all 22 patients undergoing bridging LC, compared to the 46.2% rate of one-year mortality of the 26 patients in the definitive PC cohort. One recent study in 2022 demonstrated a similar low one-year mortality at 5.2% (two patients) for PC patients bridged to LC, and a 40% mortality (20 patients) in definitive PC [23]. It is important to note as that a large proportion of the 0% mortality bridging LC cohort would be self-selecting patients who survive the 30-day mortality mark as only three patients had a delayed LC before 30 days.

Our study also demonstrated that both the mean ASA and CCI scores were statistically significantly different between the definitive PC (ASA 3.04, CCI 6.3) and bridging LC cohorts (ASA 2.61, CCI 4.39). The 2022 study mentioned EARLIER demonstrated similar findings of statistically significant differences between definitive PC (ASA 3.36, CCI 7.15), and bridging LC cohorts (ASA 2.97, CCI 6.35) [23]. This result suggests ASA and CCI can be effective predictive parameters to use when considering post-PC patients for surgery.

The article "Outcome Predictors of Percutaneous Cholecystostomy As Definitive Versus Bridging Treatment for Acute Cholecystitis" was published in 2023. Journal: Cureus.

Our study also showed that the presence of negative predictive factors of respiratory dysfunction and jaundice had significantly higher 30-day mortality and 90-day mortality rates of 31.3% and 37.5%, compared to the absence thereof at 9.4% and 21.4%, respectively. Additionally, the mean ASA was significantly lower in the one-year survival cohort (ASA 2.71) than the 30-day (ASA 3.25) and 90-day (ASA 3.25) mortality cohort. These findings are supported in similarity to the Tokyo Guidelines for general AC and other studies specifically looking at PC cohorts [5,23,24]. This shows negative predictive factors and ASA can be used as adjuncts to predict PC patient mortality.

The limitation of this study is its retrospective single-centre nature and small sample size. Although our primary outcome measure was mortality, future studies should also consider morbidity, patient quality of life outcomes, and cost-effectiveness between definitive and bridging PC.

## Conclusions

The current study demonstrates that PC is a safe option to treat AC with a high technical success rate and few major complications. Here, we demonstrate that PC is both commonly used and effective in treating a select group of co-morbid and unwell patients with AC as a bridging technique to receive delayed LC. Furthermore, our results indicate that ASA and CCI scores are valuable clinical adjuncts for evaluating whether post-PC patients would be suitable for LC. Additionally, high ASA scores and the presence of negative predictive factors of respiratory dysfunction and hyperbilirubinemia on presentation can serve as significant indicators of PC mortality.
